This article has been retracted.

# Associations between VDR Gene Polymorphisms and Osteoporosis Risk and Bone Mineral Density in Postmenopausal Women: A systematic review and Meta-Analysis

**DOI:** 10.1038/s41598-017-18670-7

**Published:** 2018-01-17

**Authors:** Liang Zhang, Xin Yin, Jingcheng Wang, Daolinag Xu, Yongxiang Wang, Jiandong Yang, Yuping Tao, Shengfei Zhang, Xinmin Feng, Caifeng Yan

**Affiliations:** 1 Department of Orthopedics, Northern Jiangsu People’s Hospital, Yangzhou, China; 2 Department of Orthopedics, First Affiliated Hospital of PLA General Hospital, Beijing, China; 3 Department of Nephrology, Northern Jiangsu People’s Hospital, Yangzhou, China; 4 Department of Endocrinology, Northern Jiangsu People’s Hospital, Yangzhou, China

## Abstract

Results on the relationships between vitamin D receptor (VDR) gene polymorphisms and postmenopausal osteoporosis (PMOP) susceptibility and bone mineral density (BMD) are conflicting. The aim of the study is to identify more eligible studies that calculated pooled OR and WMD with 95% CI to assess their associations. Overall, there were significant correlations between VDR *Apa*I, VDR *Fok*I and PMOP susceptibility. Subgroup analysis showed that VDR *Apa*I polymorphism significantly decreased the osteoporosis risk in Caucasian postmenopausal women. In Asian populations, VDR *Bsm*I and VDR *Fok*I were associated with an increased risk of PMOP. As to the associations between VDR polymorphisms and BMD, Caucasian PMOP women carrying the *Apa*I aa genotype were at risk of high BMD in femoral neck, and low femoral neck BMD was observed in Caucasian PMOP women with *Fok*I Ff genotype. PMOP women with the *Cdx*2 GA genotype had a lower lumbar spine BMD in overall and Caucasian populations compared with PMOP women with GG genotype. Different VDR gene polymorphisms have different impacts on PMOP risk and BMD.

## Introduction

Postmenopausal osteoporosis (PMOP) is a common metabolic bone disorder characterized by low bone mineral density (BMD) and increased fracture risks in postmenopausal women^1,2^. The pathogenesis of PMOP remains unclear^3^. In recent years, the association between genetic factors and PMOP susceptibility has been highlighted^4–7^.

Vitamin D has a wide range of biological functions, including calcium and phosphate homeostasis, skeletal metabolism and vascular function^8^. Vitamin D receptor (VDR) is the target receptor to regulate the transcription of Vitamin D, and is also thought to play a key role in cellular differentiation and proliferation^9^. Recently, VDR gene polymorphisms like VDR *Apa*I, VDR *Bsm*I, VDR *Cdx*2, VDR *Fok*I and VDR *Taq*I are getting an increasing recognition of importance as more studies have verified their significant associations with several diseases^9,10^.

More attention has been paid to the relationship between VDR gene polymorphisms and PMOP risk and BMD in postmenopausal women. Nevertheless, there are sdiscrepancies over this issue^11–14^. Although previous meta-analyses reported associations between VDR polymorphisms and osteoporosis risk, the results are conflicting^9,15,16^. To the best of our knowledge, there lacks evidence to confirm the relationship between VDR *Apa*I, VDR *Bsm*I, VDR *Cdx*2, VDR *Fok*I and VDR *Taq*I polymorphisms and osteoporosis risk in postmenopausal women. In addition, the relationship between VDR gene polymorphisms and BMD in postmenopausal women has also been widely studied, but the results are also controversial^11,17–26^. The aim of the present meta-analysis is to determine whether there is any significant association between VDR gene polymorphisms (VDR *Apa*I, VDR *Bsm*I, VDR *Cdx*2, VDR *Fok*I and VDR *Taq*I) and susceptibility to osteoporosis and BMD in postmenopausal women.

## Results

### Characteristics of the eligible studies

A total of 58 studies^11–14,17–25,27–71^ meeting the inclusion and exclusion criteria were recruited in our meta-analysis, among which 47 studies^11–14,17–20,22,23,25,27–62^ explored the relationships between VDR gene polymorphisms and PMOP susceptibility in postmenopausal women, and 26 studies^11,17,18,21–24,26–28,34,42,46,47,52,54,61,63–71^ eported the BMD value in PMOP women with various VDR genotypes. The study selection and inclusion processes are shown in Fig. 1. The general characteristics of the studies reporting the association with PMOP risk are indicated in Table 1, and the characteristics of the studies measuring BMD in PMOP women carrying VDR *Apa*I, VDR *Bsm*I, VDR *Taq*I, VDR *Cdx*2 and VDR *Fok*I polymorphisms are shown in Table 2.

**Figure 1:** The study selection and inclusion process.

**Table 1:** General characteristics of studies assciated with postmenopausal osteoporosis risk.

Author	Year	Ethnicity	Sample Size		VDR *Apa*I									
					Case					Control				
			Case	Control	A	a	AA	Aa	aa	A	a	AA	Aa	aa
Sassi *et al*.	2015	Caucasian	141	231	103	179	25	53	63	167	295	26	115	90
Castelán-Martínez *et al*.	2015	Caucasian	387	147	332	442	86	160	141	127	167	26	75	46
González-Mercado *et al*.	2013	Caucasian	88	87	99	77	26	47	15	99	75	29	41	17
Marozik *et al*.	2013	Caucasian	54	77	70	38	23	24	7	62	92	14	34	29
Yoldemir *et al*.	2011	Caucasian	130	130	128	132	34	60	36	135	125	31	73	26
Luan *et al*.	2011	Asian	77	227	93	61	42	9	26	221	233	102	17	108
Tanriover *et al*.	2010	Caucasian	50	50	53	47	15	23	12	57	43	22	13	15
Seremak-Mrozikiewicz *et al*.	2009	Caucasian	163	63	152	174	35	82	46	56	70	12	32	19
Uysal *et al*.	2008	Caucasian	100	146	120	80	35	50	15	171	121	46	79	21
Chen *et al*.	2007	Asian	82	113	24	140	4	16	62	65	161	12	41	60
Mitra *et al*.	2006	Asian	119	97	144	94	50	44	25	101	93	34	33	30
Duman *et al*.	2004	Caucasian	75	66	82	68	13	56	6	75	57	15	45	6
Douroudis *et al*.	2003	Caucasian	35	44	36	34	11	14	10	60	28	17	26	1
Zajícková *et al*.	2002	Caucasian	65	33	79	51	23	33	9	37	29	10	17	6
Langdahl *et al*.	2000	Caucasian	78	74	88	68	22	44	12	82	66	25	32	17
Gennari *et al*.	1998	Caucasian	160	144	217	103	68	81	11	152	136	34	84	26
Vandevyver *et al*.	1997	Caucasian	87	699	85	89	20	45	22	769	629	197	375	127
Riggs *et al*.	1995	Caucasian	40	128	43	37	12	19	9	135	121	38	59	31
**Author**	**Year**	**Ethnicity**	**Sample Size**		**VDR** ***Bsm*** **I**									
					**Case**					**Control**				
			**Case**	**Control**	**B**	**b**	**BB**	**Bb**	**bb**	**B**	**b**	**BB**	**Bb**	**bb**
D. Boroń *et al*.	2015	Caucasian	278	292	323	233	101	121	56	369	215	128	113	51
Marozik *et al*.	2013	Caucasian	54	77	55	53	12	31	11	48	106	11	26	40
Pouresmaeili *et al*.	2013	Caucasian	64	82	61	67	14	33	17	59	105	13	33	36
González-Mercado *et al*.	2013	Caucasian	88	88	40	136	6	28	54	46	130	4	38	46
Efesoy *et al*.	2011	Caucasian	40	30	33	47	5	23	12	25	35	5	15	10
Yoldemir *et al*.	2011	Caucasian	130	130	117	143	22	73	35	109	151	22	65	43
Tanriover *et al*.	2010	Caucasian	50	50	49	51	15	19	16	45	55	19	7	24
Mansour *et al*.	2010	Caucasian	50	20	69	31	27	15	8	4	36	1	2	17
Musumeci *et al*.	2009	Caucasian	100	200	114	86	30	54	16	133	267	15	103	82
Mencej-Bedrac *et al*.	2009	Caucasian	240	228	164	316	27	110	103	180	276	40	100	88
Seremak-Mrozikiewicz *et al*.	2009	Caucasian	163	63	120	206	27	66	70	47	79	10	27	26
Pérez *et al*.	2008	Caucasian	64	68	69	59	17	35	12	72	64	20	32	16
Uysal *et al*.	2008	Caucasian	100	146	84	116	18	48	34	126	166	24	78	44
Mitra *et al*.	2006	Asian	119	97	148	90	51	46	22	76	118	19	38	40
Duman *et al*.	2004	Caucasian	75	66	90	60	18	54	3	76	56	17	42	7
Zhu *et al*.	2004	Asian	40	158	38	42	6	26	8	119	197	7	105	46
Douroudis *et al*.	2003	Caucasian	35	44	18	52	3	12	20	49	39	10	29	5
Chen *et al*.	2003	Asian	40	21	7	73	0	7	33	3	39	0	3	18
Lisker *et al*.	2003	Caucasian	66	57	47	85	15	17	34	64	50	13	38	6
Borjas-Fajardo *et al*.	2003	Caucasian	54	55	76	32	28	20	6	58	52	11	36	8
Zajícková *et al*.	2002	Caucasian	65	33	66	64	21	24	20	33	33	10	13	10
Pollak *et al*.	2001	Asian	75	143	64	86	13	38	24	99	187	16	67	60
Aerssens *et al*.	2000	Caucasian	135	239	112	158	26	60	49	229	249	52	125	62
Langdahl *et al*.	2000	Caucasian	80	80	84	76	23	38	19	84	76	25	34	21
Garrofé *et al*.	2000	Caucasian	75	51	67	83	9	49	17	42	60	10	22	19
Poggi *et al*.	1999	Caucasian	50	225	47	53	6	35	9	47	53	63	95	67
Go´mez *et al*.	1999	Caucasian	37	122	34	40	7	20	10	91	153	20	51	51
Gennari *et al*.	1998	Caucasian	155	136	172	138	40	92	23	98	174	11	76	49
Zhang *et al*.	1998	Asian	17	162	3	31	0	3	14	14	310	0	14	148
Vandevyver *et al*.	1997	Caucasian	86	698	74	98	12	50	24	622	774	127	368	203
Houstan *et al*.	1996	Caucasian	44	44	35	53	8	19	17	37	51	9	19	16
Berg *et al*.	1996	Caucasian	19	30	16	22	4	8	7	27	33	8	11	11
Yanagi *et al*.	1996	Asian	46	66	36	56	12	12	22	11	121	2	7	57
Riggs *et al*.	1995	Caucasian	40	129	38	42	9	20	11	101	157	20	61	48
Lim *et al*.	1995	Asian	72	70	13	131	2	9	61	11	129	1	9	60
Melhus *et al*.	1994	Caucasian	70	76	57	83	14	29	27	103	49	34	35	7
**Author**	**Year**	**Ethnicity**	**Sample Size**		**VDR** ***Taq*** **I**									
					**Case**					**Control**				
			**Case**	**Control**	**T**	**t**	**TT**	**Tt**	**tt**	**T**	**t**	**TT**	**Tt**	**tt**
Ziablitsev *et al*.	2015	Caucasian	44	30	58	30	20	18	6	20	40	4	12	14
Sassi *et al*.	2015	Caucasian	141	231	173	109	58	57	26	301	161	103	95	33
González-Mercado *et al*.	2013	Caucasian	88	88	136	40	54	28	6	128	48	46	36	6
Marozik *et al*.	2013	Caucasian	54	77	60	48	17	26	11	102	52	39	24	14
Yoldemir *et al*.	2011	Caucasian	130	130	161	99	51	59	20	157	103	49	59	22
Tanriover *et al*.	2010	Caucasian	50	50	59	41	15	29	6	67	33	25	17	8
Seremak-Mrozikiewicz *et al*.	2009	Caucasian	163	63	215	111	78	59	26	73	53	22	29	12
Uysal *et al*.	2008	Caucasian	100	146	126	74	40	46	14	183	109	54	75	17
Mitra *et al*.	2006	Asian	119	97	110	128	34	42	43	119	75	44	31	22
Duman *et al*.	2004	Caucasian	75	66	88	62	23	42	10	74	58	23	28	15
Douroudis *et al*.	2003	Caucasian	35	44	51	19	19	13	3	43	45	8	27	9
Zajícková *et al*.	2002	Caucasian	65	33	77	53	23	31	11	36	30	11	14	8
Langdahl *et al*.	2000	Caucasian	78	75	87	69	23	41	14	90	60	28	34	13
Masi *et al*.	1998	Caucasian	90	111	62	118	13	36	41	82	140	9	64	38
Gennari *et al*.	1998	Caucasian	160	144	153	167	33	87	40	195	93	62	71	11
Vandevyver *et al*.	1997	Caucasian	46	284	52	40	11	30	5	341	227	91	159	34
Riggs *et al*.	1995	Caucasian	41	130	45	37	11	23	7	163	97	53	57	20
**Author**	**Year**	**Ethnicity**	**Sample Size**		**VDR** ***Cdx*** **2**									
					**Case**					**Control**				
			**Case**	**Control**	**G**	**A**	**GG**	**GA**	**AA**	**G**	**A**	**GG**	**GA**	**AA**
Marozik *et al*.	2013	Caucasian	54	77	95	13	41	13	0	130	24	53	24	0
Ziablitsev *et al*.	2015	Caucasian	44	30	52	36	16	20	8	16	44	2	12	16
Mencej-Bedrac *et al*.	2009	Caucasian	239	228	385	93	155	75	9	392	64	172	48	8
**Author**	**Year**	**Ethnicity**	**Sample Size**		**VDR** ***Fok*** **I**									
					**Case**					**Control**				
			**Case**	**Control**	**F**	**f**	**FF**	**Ff**	**ff**	**F**	**f**	**FF**	**Ff**	**ff**
Langdahl *et al*.	2000	Caucasian	79	80	97	61	28	41	10	99	61	34	31	15
Tanriover *et al*.	2010	Caucasian	50	50	76	24	27	22	1	76	24	29	18	3
Zajícková *et al*.	2002	Caucasian	65	33	80	50	26	28	11	35	31	7	21	5
Yasovanthi *et al*.	2011	Caucasian	247	254	327	167	104	119	24	368	140	122	124	8
Gennari *et al*.	1999	Caucasian	164	119	193	135	60	73	31	161	77	53	55	11
Choi *et al*.	2000	Asian	48	65	47	49	12	23	13	85	45	26	33	6
Lucotte G *et al*.	1999	Caucasian	124	105	159	89	45	69	10	132	78	40	52	13
Lisker *et al*.	2003	Caucasian	65	57	83	47	27	29	9	69	45	20	29	8
Mitra *et al*.	2006	Asian	119	97	118	120	38	42	39	125	69	46	33	18
Mansour *et al*.	2010	Caucasian	50	20	77	23	34	9	7	40	0	20	0	0
Mencej-Bedrac *et al*.	2009	Caucasian	240	228	284	196	88	108	44	307	149	105	97	26
Pérez *et al*.	2008	Caucasian	64	68	76	52	22	32	10	80	56	22	36	10
Yoldemir *et al*.	2011	Caucasian	130	130	187	73	66	55	9	179	81	62	55	13
Mohammadi *et al*.	2015	Caucasian	139	31	163	115	80	3	56	25	37	11	3	17
González-Mercado *et al*.	2013	Caucasian	88	88	98	78	25	48	15	93	83	24	45	19

**Table 2:** Characteristics of included studies of lumbar spine, femoral neck and Ward’s triangle BMD in VDR *Apa*I, VDR *Bsm*I, VDR *Taq*I, VDR *Cdx*2 and VDR *Fok*I genotypes.

VDR *Apa*I			Lumbar Spine BMD						VDR *Apa*I			Femoral Neck BMD					
			AA		Aa		aa					AA		Aa		aa	
Author	Year	Ethnicity	N	Mean ± SD	N	Mean ± SD	N	Mean ± SD	Author	Year	Ethnicity	N	Mean ± SD	N	Mean ± SD	N	Mean ± SD
Pedrera-Canal *et al*.	2015	Caucasian	85	0.74 ± 0.08	125	0.74 ± 0.07	64	0.75 ± 0.08	Marozik *et al*.	2013	Caucasian	23	0.77 ± 0.03	24	0.87 ± 0.03	7	0.86 ± 0.04
Marozik *et al*.	2013	Caucasian	23	0.91 ± 0.04	24	0.98 ± 0.03	7	1.04 ± 0.06	Horst-Sikorska *et al*.	2013	Caucasian	107	0.69 ± 0.08	295	0.69 ± 0.09	135	0.75 ± 0.09
Horst-Sikorska *et al*.	2013	Caucasian	107	0.85 ± 0.14	295	0.84 ± 0.15	135	0.85 ± 0.14	Duman *et al*.	2004	Caucasian	13	0.69 ± 0.02	56	0.69 ± 0.01		
Yoldemir *et al*.	2011	Caucasian	34	1.02 ± 0.11	60	1.00 ± 0.12	36	1.01 ± 0.12	Pedrera-Canal *et al*.	2015	Caucasian	85	0.69 ± 1.00	125	0.72 ± 0.09	64	0.71 ± 0.10
Duman *et al*.	2004	Caucasian	13	0.83 ± 0.05	56	0.79 ± 0.02			Yoldemir *et al*.	2011	Caucasian	34	0.84 ± 0.08	60	0.81 ± 0.09	36	0.87 ± 0.14
Vandevyver *et al*.	1997	Caucasian	17	0.73 ± 0.08	34	0.71 ± 0.13	14	0.67 ± 0.09									
**VDR** ***Bsm*** **I**			**Lumbar Spine BMD**						**VDR** ***Bsm*** **I**			**Femoral Neck BMD**					
			**BB**		**Bb**		**bb**					**BB**		**Bb**		**bb**	
Marozik *et al*.	2013	Caucasian	12	0.95 ± 0.06	31	0.95 ± 0.03	11	1.02 ± 0.04	Marozik *et al*.	2013	Caucasian	12	0.79 ± 0.03	31	0.84 ± 0.03	11	0.85 ± 0.03
D. Boroń *et al*.	2015	Caucasian	101	0.8 ± 0.02	121	0.83 ± 0.04	56	0.83 ± 0.06	Garrofé *et al*.	2000	Caucasian	17	0.71 ± 0.10	65	0.73 ± 0.08	23	0.76 ± 0.07
Garrofé *et al*.	2000	Caucasian	17	0.79 ± 0.04	65	0.79 ± 0.03	23	0.8 ± 0.04	Ge *et al*.	2006	Asian	5	0.65 ± 0.02	33	0.69 ± 0.07	142	0.69 ± 0.08
Poggi *et al*.	1999	Caucasian	6	0.84 ± 0.14	35	0.88 ± 0.13	9	0.91 ± 0.16	Garnero *et al*.	2005	Caucasian	90	0.80 ± 0.11	62	0.81 ± 0.12	33	0.81 ± 0.12
Ge *et al*.	2006	Asian	5	0.76 ± 0.07	33	0.73 ± 0.07	142	0.74 ± 0.09	Houstan *et al*.	1996	Caucasian	8	0.79 ± 0.04	19	0.73 ± 0.03	17	0.67 ± 0.03
Houstan *et al*.	1996	Caucasian	8	0.87 ± 0.05	19	0.89 ± 0.04	17	0.81 ± 0.04	Horst-Sikorska *et al*.	2013	Caucasian	82	0.70 ± 0.09	225	0.70 ± 0.09	193	0.69 ± 0.08
Horst-Sikorska *et al*.	2013	Caucasian	82	0.86 ± 0.15	225	0.85 ± 0.15	193	0.84 ± 0.14	Duman *et al*.	2004	Caucasian	18	0.67 ± 0.02	54	0.69 ± 0.01		
Palomba *et al*.	2005	Caucasian	208	0.62 ± 0.06	416	0.61 ± 0.06	476	0.62 ± 0.06	Aerssens *et al*.	2000	Caucasian	26	0.71 ± 0.09	60	0.69 ± 0.10	49	0.70 ± 0.09
Duman *et al*.	2004	Caucasian	18	0.84 ± 0.04	54	0.79 ± 0.02			Mencej-Bedrac *et al*.	2009	Caucasian	27	0.60 ± 0.08	110	0.64 ± 0.09	103	0.62 ± 0.08
Aerssens *et al*.	2000	Caucasian	26	1.01 ± 0.22	60	0.81 ± 0.16	49	0.87 ± 0.21	Pérez *et al*.	2008	Caucasian	16	0.60 ± 0.01	43	0.58 ± 0.01	13	0.54 ± 0.04
Palomba *et al*.	2003	Caucasian	12	0.58 ± 0.08	23	0.58 ± 0.08	29	0.57 ± 0.07	Yoldemir *et al*.	2011	Caucasian	22	0.82 ± 0.06	73	0.84 ± 0.11	35	0.84 ± 0.11
Vandevyver *et al*.	1997	Caucasian	10	0.69 ± 0.08	38	0.71 ± 0.12	17	0.72 ± 0.11	Wu *et al*.	2007	Asian	12	0.70 ± 0.07	60	0.71 ± 0.09	126	0.69 ± 0.09
Mencej-Bedrac *et al*.	2009	Caucasian	27	0.73 ± 0.09	110	0.75 ± 0.08	103	0.74 ± 0.10	Pedrera-Canal *et al*.	2015	Caucasian	107	0.69 ± 0.10	215	0.71 ± 0.06	134	0.7 ± 0.09
Pérez *et al*.	2008	Caucasian	17	0.69 ± 0.02	34	0.66 ± 0.02	13	0.67 ± 0.02	Moran *et al*.	2015	Caucasian	18	0.72 ± 0.10	65	0.70 ± 0.10	67	0.70 ± 0.09
Yoldemir *et al*.	2011	Caucasian	22	1.02 ± 0.08	73	1.02 ± 0.12	35	1.01 ± 0.13	Creatsa *et al*.	2011	Caucasian	7	0.77 ± 0.08	23	0.73 ± 0.16	12	0.66 ± 0.15
Wu *et al*.	2007	Asian	12	0.87 ± 0.09	60	0.87 ± 0.12	126	0.77 ± 0.11									
Pedrera-Canal *et al*.	2015	Caucasian	107	0.77 ± 0.07	215	0.74 ± 0.07	134	0.75 ± 0.07									
Moran *et al*.	2015	Caucasian	18	0.71 ± 0.06	65	0.72 ± 0.08	67	0.74 ± 0.06									
Creatsa *et al*.	2011	Caucasian	7	0.92 ± 0.14	23	0.85 ± 0.18	12	0.93 ± 0.17									
**VDR** ***Bsm*** **I**			**Ward’s triangle BMD**						**VDR** ***Taq*** **I**			**Femoral Neck BMD**					
			**BB**		**Bb**		**bb**					**TT**		**Tt**		**tt**	
**Author**	**Year**	**Ethnicity**	**N**	**Mean ± SD**	**N**	**Mean ± SD**	**N**	**Mean ± SD**									
Garrofé *et al*.	2000	Caucasian	17	0.58 ± 0.11	65	0.59 ± 0.09	23	0.64 ± 0.11									
Ge *et al*.	2006	Asian	5	0.50 ± 0.06	33	0.49 ± 0.08	142	0.49 ± 0.13									
Duman *et al*.	2004	Caucasian	18	0.51 ± 0.03	54	0.54 ± 0.02											
Wu *et al*.	2007	Asian	12	0.66 ± 0.09	60	0.58 ± 0.10	126	0.57 ± 0.10									
**VDR** ***Taq*** **I**			**Lumbar Spine BMD**						**VDR** ***Taq*** **I**			**Femoral Neck BMD**					
			**TT**		**Tt**		**tt**					**TT**		**Tt**		**t**	
Marozik *et al*.	2013	Caucasian	17	1.01 ± 0.03	26	0.95 ± 0.04	11	0.91 ± 0.07	Marozik *et al*.	2013	Caucasian	17	0.85 ± 0.02	26	0.84 ± 0.03	11	0.77 ± 0.03
Ziablitsev *et al*.	2015	Caucasian	24	2.16 ± 0.09	30	1.57 ± 0.01	20	1.39 ± 0.18	Horst-Sikorska *et al*.	2013	Caucasian	199	0.69 ± 0.08	218	0.7 ± 0.09	84	0.69 ± 0.09
Horst-Sikorska *et al*.	2013	Caucasian	199	0.83 ± 0.14	218	0.85 ± 0.15	84	0.87 ± 0.15	Duman *et al*.	2004	Caucasian	23	0.73 ± 0.02	42	0.68 ± 0.02	10	0.63 ± 0.03
Duman *et al*.	2004	Caucasian	23	0.87 ± 0.03	42	0.77 ± 0.02	10	0.80 ± 0.05	Yoldemir *et al*.	2011	Caucasian	51	0.86 ± 0.13	59	0.81 ± 0.08	20	0.84 ± 0.08
**VDR** ***Cdx*** **2**			**Lumbar Spine BMD**						**VDR** ***Cdx*** **2**			**Femoral Neck BMD**					
			**GG**		**GA**		**AA**					**GG**		**GA**		**AA**	
Marozik *et al*.	2013	Caucasian	41	0.96 ± 0.03	13	0.99 ± 0.04	0	0	Marozik *et al*.	2013	Caucasian	41	0.82 ± 0.02	13	0.87 ± 0.04	0	0
Ziablitsev *et al*.	2015	Caucasian	18	2.2 ± 0.14	32	1.51 ± 0.17	24	1.83 ± 0.18	Zhang *et al*.	2006	Asian	44	0.62 ± 0.02	97	0.62 ± 0.01	30	0.59 ± 0.02
Zhang *et al*.	2006	Asian	44	0.75 ± 0.03	97	0.78 ± 0.01	30	0.79 ± 0.024	Mencej-Bedrac *et al*.	2009	Caucasian	155	0.62 ± 0.08	75	0.62 ± 0.09	9	0.69 ± 0.11
Mencej-Bedrac *et al*.	2009	Caucasian	155	0.75 ± 0.09	75	0.73 ± 0.08	9	0.73 ± 0.07									
**VDR** ***Fok*** **I**			**Lumbar Spine BMD**						**VDR** ***Fok*** **I**			**Femoral Neck BMD**					
			**FF**		**Ff**		**ff**					**FF**		**Ff**		**ff**	
Yasovanthi *et al*.	2011	Caucasian	104	0.87 ± 0.12	119	0.85 ± 0.15	24	0.75 ± 0.17	Lucotte G *et al*.	1999	Caucasian	45	0.64 ± 0.12	69	0.63 ± 0.12	10	0.60 ± 0.08
Lucotte G *et al*.	1999	Caucasian	45	0.81 ± 0.15	69	0.79 ± 0.14	10	0.80 ± 0.15	Mencej-Bedrac *et al*.	2009	Caucasian	88	0.63 ± 0.08	108	0.63 ± 0.09	44	0.62 ± 0.08
Mencej-Bedrac *et al*.	2009	Caucasian	88	0.74 ± 0.09	108	0.75 ± 0.08	44	0.74 ± 0.10	Pérez *et al*.	2008	Caucasian	19	0.59 ± 0.01	33	0.58 ± 0.01	10	0.55 ± 0.02
Pérez *et al*.	2008	Caucasian	21	0.70 ± 0.02	33	0.66 ± 0.01	9	0.64 ± 0.03	Yoldemir *et al*.	2011	Caucasian	55	0.85 ± 0.11	55	0.83 ± 0.10	9	0.86 ± 0.06
Yoldemir *et al*.	2011	Caucasian	66	1.00 ± 0.12	55	1.03 ± 0.12	9	1.10 ± 0.09									
Xing *et al*.	2010	Asian	28	0.86 ± 0.09	54	0.85 ± 0.10	21	0.84 ± 0.12									

### Power analysis

Before this meta-analysis, a power analysis was conducted by using the Power and Precision V4 software to verify whether the included studies could offer adequate power (>80%). The statistical power in our study was sufficient to detect the associations between VDR gene polymorphisms and PMOP risk.

### VDR polymorphisms and PMOP risk

#### VDR *Apa*I

Overall, our study showed a significant association between VDR *Apa*I polymorphism and PMOP risk. When stratified by ethnicity, subgroup analysis indicated that there was also a significant association between VDR *Apa*I polymorphism and PMOP risk in Caucasian populations, while there lacked a significant association in Asian populations. All the data are shown in Table 3, and Fig. 2.

**Table 3:** Results of genetic models for VDR *Apa*I, VDR *Bsm*I, VDR *Taq*I, VDR *Cdx*2 and VDR *Fok*I polymorphisms and osteoporosis susceptibility in postmenopausal women.

Comparison	N	Test of association			Model	Test of heterogeneity		Begg’s test	Egger’s test
		OR	95% CI	*P* value		*P* value	I^2^ (%)	*P* value	*P* value
**VDR** ***Apa*** **I**									
Overall	18								
a *vs*. A		0.95	0.793–1.13	0.53	R	<0.001	69.2	0.649	0.575
aa *vs*. AA		0.84	0.61–1.15	0.271	R	<0.001	60.4	0.325	0.405
Aa *vs*. AA		0.86	0.73–1.01	0.063	F	0.091	32.4	0.13	0.075
Aa/aa *vs*. AA		**0.84**	**0.73–0.98**	**0.022**	F	0.020	45.3	0.058	0.076
aa *vs*. AA/Aa		0.93	0.70–1.23	0.609	R	<0.001	66.6	0.363	0.484
Caucasian	15								
a *vs*. A		0.94	0.80–1.12	0.505	R	0.001	61.6		
aa *vs*. AA		0.84	0.58–1.20	0.33	R	0.001	60.5		
Aa *vs*. AA		**0.84**	**0.70–0.99**	**0.042**	F	0.046	41.7		
Aa/aa *vs*. AA		**0.85**	**0.72–1.00**	**0.047**	F	0.017	48.8		
aa *vs*. AA/Aa		0.93	0.69–1.24	0.609	R	0.002	58.5		
Asian	3								
a *vs*. A		0.99	0.48–2.06	0.98	R	<0.001	69.2		
aa *vs*. AA		0.86	0.38–1.96	0.727	R	0.033	70.8		
Aa *vs*. AA		1.04	0.65–1.67	0.879	F	0.803	0		
Aa/aa *vs*. AA		0.81	0.57–1.15	0.238	F	0.163	44.8		
aa *vs*. AA/Aa		0.96	0.36–2.60	0.942	R	<0.001	88.1		
**VDR** ***Bsm*** **I**									
Overall	36								
B *vs*. b		1.21	1.00–1.46	0.052	R	<0.001	83	0.215	0.198
BB *vs*. bb		1.4	0.97–2.01	0.072	R	<0.001	79.4	0.358	0.194
Bb *vs*. bb		1.27	0.99–1.64	0.06	R	<0.001	73.4	0.505	0.409
BB/Bb *vs*. bb		**1.32**	**1.01–1.72**	**0.044**	R	<0.001	79.5	0.522	0.314
BB *vs*. Bb/bb		1.21	0.93–1.57	0.159	R	<0.001	71.9	0.202	0.107
Caucasian	29								
B *vs*. b		1.09	0.90–1.33	0.385	R	<0.001	82.4		
BB *vs*. b		1.18	0.81–1.71	0.396	R	<0.001	78.3		
Bb *vs*. bb		1.19	0.89–1.59	0.246	R	<0.001	76.8		
BB/Bb *vs*. bb		1.19	0.88–1.59	0.262	R	<0.001	80.6		
BB *vs*. Bb/bb		1.08	0.81–1.37	0.682	R	<0.001	68.9		
Asian	7								
B *vs*. b		**2.02**	**1.30–3.12**	**0.002**	R	0.005	68.1		
BB *vs*. bb		**4.16**	**2.20–7.88**	<**0.001**	R	0.207	32.1		
Bb *vs*. bb		**1.73**	**1.24–2.42**	**0.001**	R	0.455	0		
BB/Bb *vs*. bb		**2.14**	**1.34–3.42**	**0.001**	R	0.064	49.6		
BB *vs*. Bb/bb		**2.98**	**1.76–5.05**	<**0.001**	R	0.267	23.1		
**VDR** ***Taq*** **I**									
Overall	17								
t *vs*. T		1.03	0.83–1.28	0.782	R	<0.001	75.6	0.149	0.053
tt *vs*. TT		1.03	0.68–1.56	0.873	R	<0.001	69.2	0.053	0.023
Tt *vs*. TT		1.09	0.81–1.47	0.573	R	<0.001	66.7	0.484	0.363
Tt/tt *vs*. TT		1.07	0.79–1.46	0.66	R	<0.001	73	0.232	0.155
tt *vs*. Tt/TT		1.03	0.76–1.39	0.848	R	0.003	55.9	0.07	0.07
Caucasian	16								
t *vs*. T		0.99	0.79–1.24	0.944	R	<0.001	74.4		
tt *vs*. TT		0.97	0.63–1.48	0.872	R	<0.001	67.9		
Tt *vs*. TT		1.05	0.77–1.44	0.747	R	<0.001	67.5		
Tt/tt *vs*. T		1.02	0.74–1.41	0.89	R	<0.001	72.7		
tt *vs*. Tt/TT		0.98	0.71–1.34	0.888	R	0.005	54.7		
**VDR** ***Cdx*** **2**									
Caucasian	3								
A *vs*. G		0.67	0.23–1.96	0.466	R	<0.001	90.9	1	0.322
AA *vs*. GG		0.45	0.05–3.81	0.462	R	0.009	78.7	1	0.74
GA *vs*. GG		0.8	0.29–2.22	0.665	R	0.011	77.8	0.296	0.115
AA/GA *vs*. GG		0.65	0.20–2.12	0.479	R	0.002	84.1	0.296	0.01
AA *vs*. GG/GA		0.56	0.14–2.20	0.405	R	0.049	66.8	1	0.866
**VDR** ***Fok*** **I**									
Overall	15								
f *vs*. F		1.1	0.91–1.33	0.301	R	<0.001	63.3	0.621	0.615
ff *vs*. FF		1.26	0.84–1.89	0.262	R	0.001	61.4	1	0.451
Ff *vs*. FF		1.14	0.97–1.33	0.113	F	0.186	24.3	0.621	0.402
Ff/ff *vs*. FF		**1.19**	**1.03–1.38**	**0.021**	F	0.029	45.3	0.373	0.593
ff *vs*. Ff/FF		1.23	0.87–1.75	0.243	R	0.004	56.2	1	0.593
Caucasian	13								
f *vs*. F		1.02	0.85–1.23	0.844	R	0.006	57		
ff *vs*. FF		1.07	0.71–1.63	0.741	R	0.006	56.4		
Ff *vs*. FF		1.1	0.93–1.30	0.26	F	0.152	29.1		
Ff/ff *vs*. FF		1.12	0.96–1.31	0.146	F	0.06	41.2		
ff *vs*. Ff/FF		1.08	0.75–1.56	0.684	R	0.016	51.7		
Asian	2								
f *vs*. F		**1.88**	**1.38–2.58**	<**0.001**	R	0.844	0		
ff *vs*. FF		**3.05**	**1.67–5.60**	<**0.001**	R	0.408	0		
Ff *vs*. FF		1.53	0.92–2.54	0.101	F	0.971	0		
Ff/ff *vs*. FF		**1.95**	**1.23–3.08**	**0.004**	F	0.938	0		
ff *vs*. Ff/FF		**2.47**	**1.43–4.27**	**0.001**	R	0.395	0		

*R*: random effect model.

*F*: fixed effect model.

**Figure 2:** Forest plot describing the meta-analysis under the dominant model for the association between VDR *Apa*I polymorphism and the risk of PMOP (Aa/aa *vs*. AA).

#### VDR *Bsm*I

VDR *Bsm*I polymorphism was found to be significantly associated with risk of developing PMOP in the overall populations and Asian populations (Table 3 and Fig. 3). In contrast, we failed to observe any significant association between them in Caucasian populations (all *P* > 0.05).

**Figure 3:** Forest plot describing the meta-analysis under the dominant model for the association between VDR *Bsm*I polymorphism and the risk of PMOP (BB/Bb vs. bb).

#### VDR Cdx2

We failed to find any significant association between VDR *Cdx*2 polymorphism and PMOP risk in Caucasian populations (*P* > 0.05), nor could we confirm the association in overall and Asian populations as there lacked relevant studies. The data are shown in Table 3.

#### VDR *Fok*I

The random-effects OR estimated for PMOP susceptibility was 1.19 in the overall PMOP populations with VDR *Fok*I polymorphism (Table 3 and Fig. 4). A significant association was also observed between VDR *Fok*I polymorphism and PMOP risk in Asian populations, while no significant relationship was observed in Caucasian populations (all *P* > 0.05) (Table 3 and Fig. 4).

**Figure 4:** Forest plot describing the meta-analysis under the dominant model for the association between VDR *Fok*I polymorphism and the risk of PMOP (Ff/ff vs. FF).

#### VDR *Taq*I

Regarding VDR *Taq*I polymorphism, no significant relationship was observed between VDR *Taq*I polymorphism and PMOP susceptibility in the overall populations and Caucasian populations (both *P* > 0.05) (Table 3). However, we did not perform the subgroup analysis to detect the association between VDR *Taq*I and PMOP in Asian populations as only one study was been searched out and no sufficient dat could be used to draw any firm conclusions in Asians.

### VDR polymorphisms and BMD

#### VDR *Apa*I

aa genotype of VDR *Apa*I was significantly associated with increased BMD in the femoral neck; while no significant difference of BMD was observed at lumbar spine between PMOP women carrying aa genotype and AA genotype (Table 4). However, no significant difference was observed in either lumbar spine or femoral neck BMD between Caucasian PMOP women carrying Aa genotype and those carrying AA genotype (Table 4).

**Table 4:** Meta-analysis of differences of Lumbar, Femoral Neck and Ward’s triangle BMD between each genotype of VDR *Apa*I, *Bsm*I, *Taq*I, *Cdx*2 and *Fok*I polymorphism.

VDR *Apa*I	Aa *vs*. AA						aa *vs*. AA					
		Test of differences		Model	Test of heterogeneity			Test of differences		Model	Test of heterogeneity	
	N	WMD (95% CI)	*P* value		*P* value	I^2^ (%)	N	WMD (95% CI)	*P* value		*P* value	I^2^ (%)
Lumbar BMD (Caucasian)	6	−0.00 (−0.04, 0.04)	0.896	R	<0.001	90.5	5	0.01 (−0.04, 0.07)	0.571	R	<0.001	87.1
Femoral Neck BMD (Caucasian)	5	0.02 (−0.03, 0.07)	0.488	R	<0.001	96.5	4	**0.06 (0.05, 0.08)**	**<0.001**	F	0.156	42.5
VDR *Bsm*I	Bb *vs*. bb						BB *vs*. bb					
**Lumbar BMD**												
Overall	18	0.00 (−0.01, 0.02)	0.699	R	<0.001	82.9	18	0.01 (−0.01, 0.02)	0.467	R	<0.001	78
Caucasian	16	−0.00 (−0.02, 0.01)	0.684	R	<0.001	78.5	16	−0.00 (−0.02, 0.02)	0.988	R	<0.001	76
Asian	2	0.05 (−0.05, 0.14)	0.344	R	<0.001	94.4	2	0.07 (−0.01, 0.14)	0.078	R	0.068	70
**Femoral Neck BMD**												
Overall	14	0.01 (−0.00, 0.03)	0.061	R	<0.001	70.2	15	0.01 (−0.02, 0.03)	0.618	R	<0.001	89.5
Caucasian	12	0.01 (−0.00, 0.03)	0.087	R	<0.001	73.9	13	0.01 (−0.02, 0.04)	0.484	R	<0.001	90.1
Asian	2	0.01 (−0.01, 0.03)	0.43	R	0.456	0	2	−0.02 (−0.05, 0.02)	0.302	R	0.14	54
**Ward’s triangle BMD**												
Overall	3	−0.01 (−0.04, 0.03)	0.645	R	0.095	57.6	3	0.02 (−0.07, 0.10)	0.675	R	0.002	83.7
Asian	2	0.01 (−0.02, 0.03)	0.55	R	0.444	0	2	0.05 (−0.02, 0.13)	0.156	R	0.051	−73.7
VDR *Taq*I	Tt *vs*. TT						tt *vs*. TT					
Lumbar BMD (Caucasian)	6	−0.12 (−0.26, 0.03)	0.108	R	<0.001	99.4	6	−0.15 (−0.30, 0.01)	0.06	R	<0.001	98.3
Femoral Neck BMD (Caucasian)	4	−0.02 (−0.06, 0.01)	0.186	R	<0.001	93.7	4	−0.05 (−0.10, 0.00)	0.072	R	<0.001	94.4
VDR *Cdx*2	GA *vs*. GG						AA *vs*. GG					
**Lumbar BMD**												
Overall	4	−**0.15** (−**0.25**, −**0.04)**	**0.007**	R	<0.001	98.9	3	−0.11 (−0.26, 0.05)	0.176	R	<0.001	97.2
Caucasian	3	−**0.22** (−**0.43**, −**0.01)**	**0.037**	R	<0.001	99.2	2	−0.19 (−0.54, 0.15)	0.274	R	<0.001	97.5
**Femoral Neck BMD**												
Overall	3	0.02 (−0.01, 0.04)	0.229	R	0.002	84.2	2	0.01 (−0.08, 0.11)	0.776	R	0.01	84.9
Caucasian	2	0.02 (−0.02, 0.07)	0.254	R	0.011	84.5						
VDR *Fok*I	Ff *vs*. FF						ff *vs*. FF					
**Lumbar BMD**												
Overall	6	−0.01 (−0.03, 0.01)	0.342	R	0.003	71.9	6	−0.02 (−0.07, 0.03)	0.481	R	<0.001	84.9
Caucasian	5	−0.01 (−0.04, 0.02)	0.444	R	0.001	77.2	5	−0.02 (−0.08, 0.04)	0.584	R	<0.001	87.9
Femoral Neck BMD (Caucasian)	4	−**0.02** (−**0.02**, −**0.01)**	**<0.001**	F	0.626	0	4	−0.02 (−0.05, 0.01)	0.149	R	0.016	71.1

*R*: random effect model.

*F*: fixed effect model.

#### VDR *Bsm*I

No significant difference of Ward’s triangle BMD was observed between the Bb genotype and bb genotype in Asian and overall populations (both *P* > 0.05) (Table 4). In addition, we failed to observe any significant difference in lumbar spine BMD and femoral neck BMD between Bb and bb genotypes in either overall, Caucasian or Asian PMOP populations (all *P* > 0.05). As shown in Table 4, there was no significant difference in lumbar spine BMD, femoral neck BMD and Ward’s triangle BMD between Caucasian and Asian PMOP women with BB genotype and those with bb genotype (all *P* > 0.05).

#### VDR Cdx2

Among PMOP women with VDR *Cdx*2 polymorphism, the GA genotype was significantly associated with reduced lumbar spine BMD in overall and Caucasian populations, but no significant difference was observed in the femoral neck (all *P* > 0.05). In addition, VDR *Cdx*2 was also not significantly associated with BMD in lumbar spine and BMD in femoral neck in etither overall populations. All the data are shown in Table 4.

#### VDR *Fok*I

The femoral neck BMD in Caucasian PMOP women with VDR *Fok*I Ff genotype was significantly lower than that in women with VDR *Fok*I FF genotype, while no significant difference was observed in lumbar spine BMD in either overall and Caucasian populations (Table 4). The VDR *Fok*I ff genotype was not significantly associated with BMD of the lumbar spine and femoral neck in PMOP women (all *P* > 0.05).

#### VDR *Taq*I

No significant difference was observed in lumbar spine BMD and femoral neck BMD between Caucasian PMOP women carrying VDR *Taq*I Tt, VDR *Taq*I tt and VDR *Taq*I TT genotypes (all *P* > 0.05) (Table 4).

### Sensitivity analysis and publication bias

We performed a leave-one-out analysis, and any single study could be omitted, without any effect on the overall statistical significance, indicating that the results were stable. The Begg’s and Egger’s tests were performed and the results indicated that there was minimal evidence of publication bias. The shape of funnel plot was symmetrical, which also indicated that there was no publication bias in our study (Fig. 5).

**Figure 5:** Funnel plot of the VDR gene polymorphism and PMOP risk.

## Discussion

### VDR *Apa*I polymorphism and risk of PMOP and BMD

VDR *Apa*I polymorphism is located in the 3′-regulatory region of VDR gene (in intron 8), resulting in changes of biological functions of Vitamin D^31^. Overall, VDR *Apa*I polymorphism has a protective effect against the development of PMOP in the overall populations and Caucasian populations, suggesting that postmenopausal women with VDR *Apa*I mutant might have less opportunity to suffer from PMOP compared with wide genotypes, which is consistent with many other studies^27,31,41^. However, controversial results were reported in Douroudis’s study^40^. In addition, the meta-analysis by Zintzaras *et al*.^15^ reported that the allele contrast for Caucasian populations showed no association for *Apa*I, which is inconsistent with our finding. When we compared our study with this study^15^, we could find that several studies^12,27,31–39^ performed after the publication year of it^15^ were searched out and included in our pooled analysis, suggesting that our meta-analysis could provide a more precise evaluation of the relationship between VDR *Apa*I polymorphism and PMOP risk.

In our study, we found that the aa genotype of VDR *Apa*I was significantly associated with increased BMD in the femoral neck, which is consistent with some studies^21,27^. However, no significant difference in BMD was observed at the lumbar spine, which is consistent with three case-control studies^21,24,34^. Marozik *et al*.^27^ reported a significant association between VDR *Apa*I polymorphism and lumbar spine BMD in PMOP women, and in their opinion, VDR *Apa*I polymorphism might be a useful marker for osteoporosis screening at least in Belarusian women. VDR *Apa*I polymorphism is found in the non-coding region of the VDR gene and may have no significant effect on the final protein product; therefore, why there are controversial results in lumbar spine and femoral neck BMD needs to be further studied. In addition, no significant difference was observed in either lumbar spine or femoral neck BMD between Caucasian PMOP women carrying Aa genotype and those carrying AA genotype, suggesting that different genotypes might have different effects on BMD.

### VDR *Bsm*I polymorphism and risk of PMOP and BMD

VDR *Bsm*I is located in the 3′ untranslated region, and involved in regulating the stability of VDR mRNA. Our study showed that VDR *Bsm*I was significantly associated with the increased risk of developing PMOP in the overall populations as well as Asian populations, which is consistent with three previous studies^39,48,56^. In contrast, no association was observed in some other studies^49,51,53,57^. The combination of different original data in each study might have great impact on the pooled distribution of each genotype, which might be an important contributor to the different results of our results and other studies. Our results are consistent with Jia *et al*.^16^ and Zintzaras *et al*.’s study^15^. However, no significant association was observed in Asian populations in other studies^8,9,16^. As Qin *et al*.^9^ included all the osteoporotic patients, and Zhao *et al*.^8^ only analyzed three studies, our study may provide a more precise evaluation than theirs. As no significant association was observed between VDR *Bsm*I and PMOP risk in Caucasian populations, ethnicity might be a factor contributing to this difference with Asian populations.

We compared BMD at the lumbar spine, femoral neck or Ward’s triangle in PMOP women with BB, Bb and bb genotypes, and found that PMOP women carrying Bb genotype or BB genotype were not at a significantly higher risk of low BMD at lumbar spine, femoral neck, and Ward’s triangle than those carrying bb genotype. As VDR *Bsm*I may not affect the amino acid sequence of VDR, it is easily understood that *Bsm*I Bb and BB genotype might not play a key role in BMD at lumbar spine, femoral neck, and Ward’s triangle. Two studies^72,73^ found no relationship between VDR *Bsm*I polymorphism and fracture risk in PMOP women, which verifies our results on the other hand.

Interestingly, our results showed consistency: VDR *Apa*I was associated with a decreased risk of PMOP, and high levels of BMD, whereas *Bsm*I was associated with an increased risk of PMOP and did not play a key role in BMD. Theoretically, the consistent results should be observed in the subgroup analysis, for both VDR *Apa*I and VDR *Bsm*I have influences on the stability of VDR mRNA. However, different gene locations of VDR *Apa*I and VDR *Bsm*I may lead to different biological functions. Thus, the different role of VDR *Apa*I and VDR *Bsm*I in the etiology and pathogenesis of PMOP and BMD may be an important contributor to the controversial findings in our study. However, the exact mechanism of the VDR *Apa*I and VDR *Bsm*I polymorphism requires further investigation.

### VDR *Cdx*2 polymorphism and risk of PMOP and BMD

VDR *Cdx*2 polymorphism is located in the promoter region of VDR gene, which is considered to be associated with the level of calcium absorption and the receptor’s activation to Vitamin D. It was found that VDR *Cdx*2 was not significantly associated with PMOP risk in Caucasian populations, which is consistent with the finding of Marozik *et al*.^27^. One previous study^28^ showed that VDR *Cdx*2 played a protective role against the risk of PMOP, which is inconsistent with the result reported by Mencej-Bedrac *et al*.^46^, while 74 postmenopausal women were examined in the study of Ziablitsev *et al*.^28^, which might contribute to this difference.

We found that GA genotype of VDR *Cdx*2 had an increased risk of developing low BMD at the lumbar spine in overall and Caucasian populations compared with GG genotype. In addition, no significant association was observed at femoral neck BMD, which is consistent with Marozik *et al*.’s study^27^ and inconsistent with other two studies^28,46^. As to the AA genotype of VDR *Cdx*2, no significant difference in lumar BMD or femoral neck BMD was observed between PMOP women with AA genotype and those with GG genotype in either overall or Caucasian populations. In Mencej-Bedrac *et al*.’s study^46^, they observed an association between the *Cdx*2 polymorphism and vertebral fracture risk; therefore, large sample-size studies are required before a more convincing conclusion can be made.

### VDR *Fok*I polymorphism and risk of PMOP and BMD

VDR *Fok*I is a polymorphism of VDR near the 50-UTR region of the gene within the DNA-binding domain, and plays an essential role in message stability and post transcriptional processes^74^. In our meta-analysis, VDR *Fok*I was significantly associated with higher risk of developing PMOP in overall and Asian populations, but not in Caucasian populations, which is inconsistent with Zintzaras *et al*.’s meta-analysis^15^.

Our analysis indicated that the Ff genotype of VDR *Fok*I was significantly associated with decreased BMD in the femoral neck in Caucasian populations, but not in the lumbar spine. Besides, we did not observe overall associations between VDR *Fok*I and BMD in either lumbar spine or femoral neck in either overall populations or Caucasian populations with ff genotype in our meta-analysis. A study performed by Wang *et al*.^75^ showed that VDR *Fok*I was associated with BMD in postmenopausal Asian women, and could probably be used with other genetic markers together to identify individuals at high risk of osteoporosis. However, we could not make a certain conclusion whether VDR *Fok*I plays a key role in BMD value in Asians since no available data could be used in meta-analysis. Four studies^34,46,47,61^ found by our searching terms were not included in Wang’s study. In addition, we excluded three studies^39,60,76^ that were recruited in Wang’s study, because no sufficient data could be collected in their original articles.

### VDR *Taq*I polymorphism and risk of PMOP and BMD

Unlike VDR *Bsm*I, VDR *Taq*I has been proved to affect mRNA stability, leading to altered protein levels and biological functions of Vitamin D. In our study, there was no significant association in overall and Caucasian populations, which was consistent with Zintzaras *et al*.’s study^15^. More studies were included in our study compared with their study^15^, suggesting that our study might provide a more precise evaluation of the relationship between VDR *Taq*I and PMOP risk. In addition, we also did not find any significant difference in lumbar spine BMD or femoral neck BMD in comparison with PNOP women with TT, Tt and tt genotypes, which is inconsistent with two studies^22,27^. As our meta-analysis had larger sample sizes and higher statistical power, it provided a more precise evaluation of this association.

Futhermore, we should pay more attention to the implications of our results on public health and clinical practice. First, taking into consideration a significant association between VDR *Apa*I, VDR *Bsm*I, VDR *Fok*I and VDR *Taq*I and PMOP risk in different ethnicities, a conclusion might be drawn that these polymorphisms may be useful markers for osteoporosis screening in certain ethnicities. Second, screening of these genetic markers may enable an early identification of risk groups to perform preventive measures in a timely manner and also to improve treatment effectiveness, avoid complications, reduce disability and mortality rates in these patients, as well as cut down the treatment costs. Third, some more reports have confirmed the genetic background of BMD^18^. Therefore, our results could provide theories that these VDR gene polymorphisms may be potential targets for genetic therapy of PMOP.

Our meta-analysis has some limitations that should be addressed. First, it should be remembered that in many cases it is the environmental factor that determines the development of PMOP. We should also remember that the absence of control for confounders such as smoking is one of the main limitations of our work because phenotypes of many diseases may be the results of interactions between genotyps and environmental factors. Second, no studies that explored the association between VDR *Apa*I, *Taq*I polymorphism and BMD in Asian populations, between VDR *Cdx*2 and PMOP risk in Asian populations have been found. Mendelian randomization (MR) study is a method of using measured variation in genes of known function to examine the causal effect of a modifiable exposure on disease in non-experimental studies. We had planned to perform MR study to reinforce the findings of our meta-analysis. However, convicing evidence in the literature cannot be provided to support the MR criteria.

In conclusion, VDR gene polymorphisms play keys roles in osteoporosis susceptibility and BMD in postmenopausal women, although different VDR gene polymorphisms might have significantly different influences on the risk of osteoporosis and BMD in PMOP women with various ethnicities.

## Materials and Methods

### Literature search

Databases including PubMed, EMBASE, Web of Science, the Cochrane Library and China WeiPu Library were searched to identify case-control studies investigating the relationship between VDR gene polymorphisms and susceptibility to PMOP and BMD. The following search terms were used to find out eligible studies exploring the PMOP risk in postmenopausal women: (‘PMOP’ OR ‘Postmenopausal osteoporosis’ OR ‘Postmenopausal’) AND (‘VDR’ OR ‘vitamin D receptor’) AND (‘polymorphism’ OR ‘single nucleotide polymorphism’ OR ‘SNP’ OR ‘variation’). To analyze to pooled effects of VDR gene polymorphisms on BMD in postmenopausal women, we used the following search terms to find out eligible studies: ‘PMOP’ OR ‘Postmenopausal osteoporosis’ OR ‘Postmenopausal’) AND (‘VDR’ OR ‘vitamin D receptor’) AND (‘polymorphism’ OR ‘single nucleotide polymorphism’ OR ‘SNP’ OR ‘variation’) AND (‘BMD’ OR ‘bone mineral density’). Then, one-by-one screening was performed by two authors according the inclusion and exclusion criteria. No language restrictions were applied. Secondary searches of eligible studies were conducted by searching the reference lists of the selected studies, reviews or comments.

### Inclusion and exclusion criteria

The inclusion criteria of our meta-analysis were as follows: (1) case-control studies; (2) postmenopausal women with PMOP as case populations, and postmenopausal women without PMOP or healthy women as controls; (3) studies evaluating PMOP risk, alleles and genotypes of at least one of the VDR gene polymorphisms; (3) studies providing the sample size, mean and standard deviation of BMD at lumbar spine, femoral neck or Ward’s triangle in PMOP women with at least one of the VDR genotypes; (4) studies providing sufficient data (alleles and genotypes of at least one of the VDR gene polymorphisms, and BMD evaluated in cases and controls with at least one of the VDR gene polymorphisms).

The exclusion criteria were: (1) reviews or case reports that were not case-control studies; (2) studies without reporting currently available data; (3) duplicated reports.

### Data extraction

Data from the eligible studies were extracted according to the inclusion and exclusion criteria by two authors, and a consensus was reached by discussion if the researchers disagreed. In the study of associations between VDR gene polymorphisms and PMOP risk, the following data were collected: author list, year of publication, ethnicity, sample size, and allele and genotype of each gene polymorphism. In the analysis of difference in BMD in PMOP women with various VDR genotypes, we collected the following data: author list, year of publication, ethnicity, the number of cases, and BMD values of the femoral neck, lumbar spine or Ward’s triangle in each VDR genotype in PMOP women.

### Data synthesis and statistical analysis

Odds ratios (OR) and 95% confidence interval (CI) were calculated to evaluate the association between VDR gene polymorphisms and PMOP. The strength of association between VDR gene polymorphisms and PMOP susceptibility was evaluated by OR and 95% CI under the allele contrast model, heterozygote model, homozygote model and dominant model. Regarding the associations between BMD and VDR gene polymorphisms, we compared BMD in PMOP women under heterozygote and homozygote models by using the weight mean difference (WMD) and 95% CI. Power analysis was performed using the Power and Precision V4 software (Biostat Inc, Englewood, USA). The heterogeneity of included studies was examined by a chi-squared-based Q statistical test and quantified by I^2^ metric value. If I^2^ value was >50% or *P* < 0.10, ORs were pooled by the random-effects model; otherwise, the fixed-effects model was used. Sensitivity analysis was performed to assess the impact of each study on the combined effect of the present meta-analysis, and subgroup analysis was also performed according to the ethnicity of the study populations. RevMan 5.3 software was used and a P < 0.05 was considered as statistically significant.

### Data availability

All data analyzed during this study are included in this published article (and its Supplementary Information files).
